# Design of Growth Trend Map of Children and Adolescents Based on Bone Age

**DOI:** 10.1155/2022/1325061

**Published:** 2022-06-10

**Authors:** Kaiyan Chen, Weiyuan Shi, Keji Mao, Wenxiu He, Ahmedin M. Ahmed, Kai Fang

**Affiliations:** ^1^College of Computer Science and Technology, Zhejiang University of Technology, Hangzhou, China; ^2^College of Zhijiang, Zhejiang University of Technology, Shaoxing, China; ^3^Florida International University, Miami, FL, USA; ^4^College of Electrical and Information Engineering, Quzhou University, Quzhou, Zhejiang 324000, China; ^5^Faculty of Information Technology, Macau University of Science and Technology, Macau 999078, China

## Abstract

Accurate height prediction has important reference significance for the development of children and adolescents and the selection of athletes. The current mainstream height prediction methods include the B-P (Bayley–Pinneau) method and the TW2 (Tanner–Whitehouse) method. A large number of documents show that the B-P method and the TW2 method have relatively large deviations in the lifelong height prediction results of Chinese children and adolescents. Based on the data collected by the Chinese Adolescent Students' Physical Fitness and Growth and Development Health Project in Zhejiang's primary and secondary schools, this paper proposes a graph of height growth trends based on bone age. The height map of age has more reference value. Aiming at the feasibility of the height data in the statistical results, the interpolation prediction method is used to verify the data, and the height growth trend graph is drawn through the method of fitting. Validation results with actual data show that the average error of the lifetime height prediction of the height growth trend map proposed in this paper is 2.1 cm, which is 1.4 cm lower than the 3.5 cm error predicted by the B-P method and 0.4 cm lower than the 2.5 cm error predicted by the TW2 method.

## 1. Introduction

In recent years, the growth and development of children and adolescents have received widespread attention, especially the lifelong height of adulthood has effectively affected the future lives of children and adolescents. The National Nutrition Plan issued by the State Council in 2017 clearly stated that the stunting rate of Chinese children and adolescents should be kept below 5% by 2020 to promote the improvement of the national fitness [1]. Predicting the lifelong height of children and adolescents in adulthood can not only promptly intervene in the abnormal conditions of their growth and development stages but also have a positive guiding role in the cultivation of life habits during the growth of children and adolescents. Therefore, proposing a more accurate height prediction model has important social significance.

There are difficulties in height prediction research, such as few public data and long-term observation and verification results. At present, there is no unified prediction program in China [2]. The growth and development of children and adolescents are jointly affected by genetic factors and environmental factors. Among them, bone age is closely related to the growth and development of children and adolescents and can objectively express the growth and growth potential of children and adolescents [3]. In response to the above problems, this study conducted a large number of data samples collected through the physical health test of primary and middle school students in Zhejiang Province and the continuous observation samples provided by the Zhejiang Bone Age Research Center to study the lifelong high prediction of children and adolescents in adulthood. This research is based on the factor that the height growth trend graph of skeletal age is used to predict the health of children and adolescents by drawing the height growth trend graph.

## 2. Research Status

The simplest method for height prediction is the genetic height calculation method proposed by Luo in Sweden [4], which predicts the height of children through the height of parents. Due to the continuous improvement of the growth samples of children and adolescents [5], the calculation formula is also constantly changing. In addition to genetic factors, the influence of acquired environment on growth and development accounts for up to 30%. Therefore, the height of children and adolescents is predicted based on the height of parents, and the error range is very large.

The GP Atlas method [6] was developed by William Walter Greulich and S. Idell Pyle of Stanford University in 1955 based on more than 7,000 wrist X-rays of healthy children from European descent families in the Cleveland area of the United States cross-tracked from 1931 to 1946. This method only needs to compare the difference between the photographed bone age film and the standard bone age film to obtain the result, and the operation is relatively simple.

Nancy Bayley of the University of California in the United States combined the GP Atlas method [6] bone age standard to propose the BP height prediction method [7]. The development types of children and adolescents are divided into early growth type, intermediate type, and delayed type. High lifetime ratio.

Tanner proposed the TW height prediction method [8] based on the bone age standard of the TW2 [9] method, which is compiled according to different genders, different ages, and different amounts of information (with or without menarche, with or without height growth, and with or without year bone age growth) and a series of multiple regression models [10]. Because the number of samples tracked and observed by this method is only 600 men and women, the data are not evenly distributed across all ages, so the prediction error is relatively large, especially for children and adolescents with early development. The prediction results are significantly higher.

The length of the human skeleton affects the growth and height of children and adolescents. Wang Yaxuan et al. [11] used samples from Yunnan province in China as experimental subjects to analyse the relationship between six body indicators, namely, hand length, foot length, hand width, foot width, inter- and intra-epicondylar humerus diameter and inter- and intra-epicondylar femur diameter, and height, to calculate the coefficients related to body indicators and height and establish the corresponding equations. Rosario et al. [12] measured body indicators such as height, weight, ulna, and arm span in children and adolescents. The Bland–Altman [13] method was used to analyse the differences and consistency between observed and predicted height.

The Capital Institute of Pediatrics of China, based on the analysis of the distribution of children's age and height data, proposed an age-based height map and height prediction curve method, which is widely used in the comparison of children's growth and development and the preliminary screening of individuals with abnormal development. Jiao Huiyong et al. used SNP sites in European DNA sequences to predict height [14] and tested Shandong Han men. The accuracy and feasibility of the experimental results are in the research stage. Zhi Yusheng et al. [15] also screened and used 22 height-associated SNP loci from a genetic perspective to construct a height prediction model and validated it in 1220 samples from northern and southern China. The feasibility of the results needs further study, and the accuracy of the model could be further improved if more SNP loci that are closely associated with height in the Chinese population can be found.

Tim J Cole proposed the Super Imposition By Translation And Rotation (SITAR) model [16] for describing adolescent growth trends in conjunction with a nonlinear mixed effects model, which introduces three variables to fit growth trends for each observer. Building on the ideas of the SITAR model, Nierop et al. proposed the QEPS (Quadratic-Exponential-Puberty-Stop) model [17], which describes the total pattern of height growth from fetus to adulthood through four basic growth functions (Q is for the quadratic function, *E* is for the exponential function, P is for the pubertal nonlinear function, and S is for the stopping growth function) and provides six modifiable parameters to describe an individual's height growth curve.

The concept of bone age [18] was put forward after X-ray was invented. It is a scale used to objectively evaluate the maturity of biological development by observing the morphology of the wrist bones [19]. Since it represents the age of the bones, and the length of the human body depends on the length of the bones, the change of bone age is closely related to the growth of height, and height prediction based on bone age is more accurate [20]. This study established a graph of height growth trends based on bone age.

## 3. Data Sample

### 3.1. Data Collection

Through the Physical Fitness and Growth and Development Health Project of Chinese Young Students, we have collected more than 90,000 pieces of data on height and bone age. A total of 24,500 primary and middle school students were selected from the overall sample, including 12,993 boys and 11,727 girls, as samples for statistical research. At the same time, 400 people who had undergone bone age assessment and are now adults were obtained from the Zhejiang Provincial Bone Age Research Center to conduct a return visit to the lifelong height after adulthood to verify the experimental results. Samples drawn from various schools in Zhejiang Province ensure that the health status of the data is better than the data collected from hospitals, and the detection data of urban and rural schools are merged for processing, and an overall average level can be obtained.

### 3.2. Statistics

When verifying the distribution of height, in order to facilitate statistics and expand the influence of individual height, the individual height is rounded up and then statistically calculated. The statistical range of boys' skeletal age starts from 6.0 years to skeletal age 18.0 years, which is the same as the statistical method of Chinese children and adolescents' age and height maps. The span of skeletal age is 0.5 years old. The statistical range of females starts from 5.5 years of bone age to 17.5 years of bone age, with 0.5 years of age as the interval. Among them, the 7-year-old bone age group corresponds to the sample data of 7.0 years old and less than 7.5 years old.

In view of the uneven dispersion of the data set, the percentile statistics method is used to calculate the data distribution [21]. Percentile statistics is to arrange a set of data from small to large and calculate the corresponding cumulative percentile. The value of any percentile is called the percentile of the percentile. The result of percentile measurement is not necessarily the center position of the interval, but it can determine the position of a value in the sample set. Percentile statistics can be used to summarize objective laws when the data sample is limited, so it is widely used [22–24].

Because the nature of percentile statistics does not require centralized representation of the data distribution, the height of each individual is included as an impact factor. The statistics of bone age are still divided by 0.5 years. Statistics on the 3rd, 25th, 50th, 75th, 97th, five percentile data, and the statistical results of male and female students are shown in Tables 1 and 2.

### 3.3. Data Verification

In order to demonstrate the feasibility of the percentile table, the above-mentioned statistical percentile table was verified. The growth and development of children and adolescents is not a linear growth process, so the height of each bone age cannot be verified by equal division. It is known that the growth of bone age tends to be gentle after 14 years old. Therefore, taking the bone age of 14 years as the boundary, the period before the bone age of 14 years is called the rapid growth and development period, and the bone age after 14 years is called the slow growth and development period, and they are verified separately. A cubic spline interpolation prediction algorithm is proposed for this, and the steps are as follows:

Step 1: the cubic spline interpolation method [25–27] can determine a polynomial of two adjacent data points through continuous data point calculation and ensure that they are continuous at the connection points. The function expression is as follows:

(1) $$\begin{array}{c} s_{i}\left(x\right)=a_{i}+\;b_{i}\left(x-x_{i}\right)+c_{i}{\left(x-x_{i}\right)}^{2}+d_{i}{\left(x-x_{i}\right)}^{3}, \end{array}$$

where *x*_*i*_ represents a certain bone age value, *a*_*i*_ represents the height value corresponding to that bone age value, and *b*_*i*_, *c*_*i*_, and *d*_*i*_ represent the coefficients of the requested polynomial.

The cubic spline interpolation method needs to determine the boundary conditions of the interpolation during the calculation process. Different boundary conditions have different interpolation methods. Since the bone age reaches the end point, there will be no height change after the epiphyseal line is completely closed, so set the end point condition to free boundary, and do not want any external force that makes the curve bend at the end point. Derive the solution of cubic spline interpolation, where is the second derivative of the node.

(2) $$\begin{array}{c} \left[\begin{array}{cccc} -h_{1} & h_{0}+h_{1} & -h_{0} & 0\\ h_{0} & 2\left(h_{0}+h_{1}\right) & h_{1} & 0\\ 0 & h_{1} & 2\left(h_{1}+h_{2}\right) & h_{2}\\ 0 & -h_{2} & \left(h_{1}+h_{2}\right) & -h_{1} \end{array}\right]\left[\begin{array}{c} m_{0}\\ m_{1}\\ \begin{array}{c} m_{2}\\ m_{3} \end{array} \end{array}\right]=6\left[\begin{array}{c} \begin{array}{c} 0\\ \frac{y_{2}-y_{1}}{h_{1}}-\frac{y_{1}-y_{0}}{h_{0}} \end{array}\\ \frac{y_{3}-y_{2}}{h_{2}}-\frac{y_{2}-y_{1}}{h_{1}}\\ 0 \end{array}\right], \end{array}$$

where *h*_*i*_=*x*_*i*+1_ − *x*_*i*_ and *m*_*i*_ represents the second-order derivative of the node.

Step 2: take the 50th percentile statistics of boys as an example. In the rapid growth and development period, the heights of 7 year old, 8 year old, 9 year old, and 10 year old were 121.4 cm, 126.4 cm, 133.1 cm, and 137.4 cm, respectively. In the period of slow growth and development, the bone ages of 14 years, 15 years, 16 years, and 18 years were taken to be 161.7 cm, 168.5 cm, 172.1 cm, and 174.1 cm, respectively. Substitute into equation (2) respectively as shown below:

(3) $$\begin{array}{c} S_{1}\left(x\right)=\left\{\begin{array}{c} 121.4+b_{1}\left(x-7\right)+c_{1}{\left(x-7\right)}^{2}+d_{1}{\left(x-7\right)}^{3}\;x\in \left[7,\;8\right]\\ 126.4+b_{2}\left(x-8\right)+c_{2}{\left(x-8\right)}^{2}+d_{2}{\left(x-8\right)}^{3}\;x\in \left[8,\;9\right]\\ 133.1+b_{3}\left(x-9\right)+c_{3}{\left(x-9\right)}^{2}+d_{3}{\left(x-9\right)}^{3}\;x\in \left[9,10\right] \end{array}\right.,\\ \;S_{2}\left(x\right)=\left\{\begin{array}{c} 161.7+b_{1}\left(x-14\right)+c_{1}{\left(x-14\right)}^{2}+d_{1}{\left(x-14\right)}^{3}\;x\in \left[14,\;15\right]\\ 168.5+{}_{b}\left(x-15\right)+c_{2}{\left(x-15\right)}^{2}+d_{2}{\left(x-15\right)}^{3}\;x\in \left[15,\;16\right]\\ 172.1+b_{3}\left(x-16\right)+c_{3}{\left(x-16\right)}^{2}+d_{3}{\left(x-16\right)}^{3}\;x\in \left[16,18\right]. \end{array}\right. \end{array}$$

Solve the equation through the derived formula, and get the result.

(4) $$\begin{array}{c} S_{1}\left(x\right)=\left\{\begin{array}{c} 121.4+4.7417\left(x-7\right)+0.35{\left(x-7\right)}^{2}-0.0917{\left(x-7\right)}^{3}\;x\in \left[7,\;8\right]\\ 126.4+6.7167\left(x-8\right)+0.075{\left(x-8\right)}^{2}-0.0916{\left(x-8\right)}^{3}\;x\in \left[8,\;9\right].\\ 133.1+4.5917\left(x-9\right)-0.2{\left(x-9\right)}^{2}-0.0917{\left(x-9\right)}^{3}\;x\in \left[9,10\right] \end{array}\right.. \end{array}$$

(5) $$\begin{array}{c} S_{2}\left(x\right)=\left\{\begin{array}{c} 161.7+7.5217\left(x-14\right)-0.0001{\left(x-14\right)}^{2}-0.7217{\left(x-14\right)}^{3}\;x\in \left[14,\;15\right]\\ 168.5+5.3565\left(x-15\right)-2.1652{\left(x-15\right)}^{2}+0.4087{\left(x-15\right)}^{3}\;x\in \left[15,\;16\right].\\ 172.1+2.2522\left(x-16\right)-0.9391{\left(x-16\right)}^{2}+0.1565{\left(x-16\right)}^{3}\;x\in \left[16,18\right] \end{array}\right.. \end{array}$$

Step 3: substituting 7.5, 8.5, and 9.5 into formula (5) to calculate the results are 123.8 cm, 129.8 cm, and 135.3 cm, respectively, which are basically consistent with the statistical results of 123.5 cm, 130.1 cm, and 135.3 cm in Table 1. Substituting 14.5 and 15.5 into formula (6), the calculated results are 166.3 cm and 170.6 cm, respectively, which are basically consistent with the statistical results of 166.7 cm and 170.2 cm in Table 1.

In summary, the percentile table of this data set is extremely feasible, which increases the persuasiveness of the experimental results.

## 4. Fitting the Height Growth Trend Map

### 4.1. Fitting Curve of Height Atlas

Combining the growth pattern of children and adolescents, it can be seen that the relationship between bone age and height is not linear. The uneven curve has many shortcomings in practical applications. First, it is not clear about the growth trend of children. Estimate the relationship between the various percentile curves. Therefore, in order to make the height growth map better in practice, the curve fitting method is adopted to find the appropriate curve type to fit the observation data to the map.

Since there will be errors between the calculated value of the fitting and the actual value, in order to make the fitting result most suitable for the actual data sample, the best matching function should be found to minimize the error between the two. This paper uses the least square method [28, 29] to minimize the residual sum of squares at each point between the fitted model and the actual observation results. The standard formula is as follows, which is the fitted polynomial:

(6) $$\begin{array}{c} E^{2}=\;\min\;\sum {\left[P\left(x_{i}\right)-y_{i}\right]}^{2}. \end{array}$$

The process of solving the least squares method is the process of solving. The fitting curve equation can be set as a polynomial of degree *n*, and the formula is as follows:

(7) $$\begin{array}{c} P\left(x\right)=a_{n}x^{n}+\;a_{n-1}x^{n-1}+\text{…}+a_{1}x+\;a_{0}. \end{array}$$

Converted into a matrix form and expressed as in the following equation, where *k* is the number of test case points.

(8) $$\begin{array}{c} X=\;\left[\begin{array}{ccc} \begin{array}{cc} x_{1}^{n} & x_{1}^{n-1} \end{array} & \cdots & \begin{array}{cc} x_{1} & 1 \end{array}\\ \vdots & \ddots & \vdots \\ \begin{array}{cc} x_{k}^{n} & x_{k}^{n-1} \end{array} & \cdots & \begin{array}{cc} x_{k} & 1 \end{array} \end{array}\right]. \end{array}$$

Multiply the transposed matrix on both sides of the equation at the same time and transform to get the following equation:

(9) $$\begin{array}{c} {\left(X^{T}X\right)}^{-1}X^{T}P\left(x\right)=A. \end{array}$$

The 1 to 4° polynomials were fitted to the growth trend graphs of male and female students by solving the equations.

It can be seen from Figure 1 that boys have a downward trend when fitting the quartic function, which does not conform to the growth law. It can be seen from Figure 2 that girls show a downward trend when fitting the cubic function, and when fitting the quartic function, the trend is good and conforms to the growth law. Therefore, the third-degree polynomial is used to fit the height growth trend map based on bone age for boys, and the fourth-degree polynomial is used for girls to fit the height growth trend map based on bone age for children and adolescents in Zhejiang Province as shown in Figure 3.

### 4.2. Growth Prediction Based on Trend Graph

Through a large number of samples combined with the growth and development rules, three representative trends are summarized. From Figure 3, it can be seen that the three curves are not completely parallel, and the Euclidean distance between each bone age point is not equal. The median curve is equal to 97th. The difference between the percentile curve gradually increases, and the difference between the 3rd percentile curve gradually decreases.

In order to be able to use three growth trend curves to predict the growth trend of individuals, this study designed an algorithm based on the shortest Euclidean distance fitting to predict the growth trend of individuals. First, convert the polynomial functions of the three growth trend curves of male and female students into a data model, which is used to calculate the bone age and height. Secondly, predict the future growth trend by comparing which trend point the current bone age height is closer to and predict the height of the next bone age point (the height of the trend line plus the Euclidean distance of the bone age height). Since the two trend lines change from wide to narrow or from narrow to wide, the height of the next bone age point may be closer to the other trend lines. When predicting the height of the next bone age point, it should be converted to another data model that is closer to the trend line. Finally, the height of each bone age point is calculated one by one by the Euclidean distance between the bone age and height, and the growth trend graph is formed by connection. The specific algorithm is as follows:

The height of each bone age point is calculated by the algorithm, and the points are connected by a smooth curve to draw a growth and development trend chart based on the current bone age height. The height at the age of 18 years of bone age can be used as the predicted height based on the growth and development of the group.

## 5. Result Analysis

### 5.1. Growth Trend Analysis

This article extracts individual cases from the adult height samples of children and adolescents interviewed to verify the feasibility of the graph of height growth trends based on bone age. Because the trend graphs of men and women are different, give examples of male and female students to demonstrate the algorithm, respectively. The boys and girls used in the examples and their basic growth are shown in Tables 3 and 4 including age, bone age, and height.

A boy with a bone age of 12.3 years and an age of 11.5 years, and a test height of 145 cm, will use the algorithm proposed in this article to calculate the height values of the bone age from 12.5 years to 18 years in the interval of 0.5 years. The calculated growth trend graph based on bone age is shown in Figure 4(a). The skeletal age is 12.0 years, the age is 13.5 years, and the test height is 155.8 cm for girls, and the height value of the bone age from 12.5 years to 18 years is calculated every 0.5 years. The calculated growth trend graph based on bone age is shown in Figure 4(b).

Figure 5 shows a graph of growth trends based on age. The boy's age is 11.5 years old, the test height is 145 cm, and the predicted age-based growth trend graph is shown in Figure 5(a). The girl's age is 13.5 years and the test height is 155.8 cm. The predicted age-based growth trend is shown in Figure 5(b).

As shown in Figure 4, the growth trend map based on bone age predicts that the boy's height at the age of 13.5 is 153 cm, which is 1 cm away from the actual height of 154 cm. It is predicted that the boy's lifetime height as an adult is 172.8 cm, which is only 0.2 cm away from the lifetime height of 173 cm obtained by the return visit, and the error range is within 1 cm. The predicted height of the girl when her bone age is 13.5 years is 162.8 cm, which is 1.2 cm different from the actual height of 164 cm. It is predicted that the lifetime height in adulthood is 167.5 cm, which is more than 1.5 cm compared with the lifetime height of 166 cm obtained in the return visit. Considering the error in height measurement, it is within the acceptable range. In general, the prediction effect of the growth trend graph based on bone age is more significant.

Observing Figure 5, the age-based growth trend map predicts that the boy's height at the age of 12.5 years is 157.5, while the actual height is 154 cm, a difference of 3.5 cm between the two. It is predicted that the boy's height when he reaches 18 years old is 169.3 cm, which is 3.7 cm different from the actual lifetime height of 173 cm. The prediction results of girls are more biased. The predicted height of a girl who is 14.7 years old is 157.5 cm, which is 6.5 cm different from the actual height of 164 cm. The predicted lifetime height is 158.8 cm. Compared with the actual lifetime height of 166 cm, the difference is 7.2 cm.

The test heights of the boys and girls in the test cases are close to the median curve, indicating that they are within the normal height range of the corresponding age group. The age of 18 does not mean that the bone age is mature, so there is still room for growth. Comparing the growth trend map based on bone age and the growth trend map based on age, the growth trend map based on bone age can describe the growth trend more accurately, and the predicted result is more accurate.

### 5.2. Comparative Analysis of Lifetime Height

The comparison results of the growth trend prediction based on bone age and the growth trend prediction based on age are shown in Figure 6, where the abscissa represents the development progress of the tested children and adolescents from the detection period, with years as the unit, and the ordinate represents the predicted height in the future. The age increases with the passage of time, while the increase of bone age may remain the same for a period of time due to objective factors, and the growth rate is not uniform. With the increase of age, the bone age may not increase simultaneously. In Figure 6(a), because the bone age of the test boy is greater than the age, the height prediction based on the bone age in the comparison chart ends early. The bone age reaching 18 years indicates the end of bone closure growth and development, and the height result is close to the actual lifetime height. The age-based growth trend shows a steady trend at the end of the curve, but in fact, there is still growth, which is slightly inconsistent with the development process. Because the test girls are older than the bone age, the height prediction based on age in the comparison chart ends early. It is observed that the difference between the predicted result based on age and the actual result is up to 7 cm, and the growth trend chart shows that the development potential is limited, and the probability of rapid growth is small. According to the comparison results of the two, the growth trend based on bone age has more reference value than the growth trend based on age.

The age-based height growth trend map predicts that there is a big gap between the height at the age of 18 and the lifetime height after adulthood. Explained from the perspective of growth and development, it shows that reaching 18 years of age is not the end of development. It can continue to grow. It is more objective to see whether the development is completed and whether the bones are closed. From the perspective of the use of the map, it shows that the growth trend prediction of children and adolescents based on the currently recognized age-based height growth trend map is not applicable, and there are large errors.

Use the continuous observation sample provided by Zhejiang Bone Age Research Center to verify the height of 400 children and adolescents from the perspective of group growth through the height growth trend map based on bone age. The average error is 2.1 cm, which is higher than the B-P method. The 3.5 cm error of the obtained height is 1.4 cm lower than the 2.5 cm error of the height predicted by the TW2 method by 0.4 cm.

## 6. Conclusions and Prospects

In this paper, through the statistical analysis of the data on the physical health of the primary and middle school students in Zhejiang Province, the interpolation prediction method is used to verify the feasibility of the data, and the least square method is used to curve the results to plot the height growth trend of children and adolescents in Zhejiang Province based on the bone age. The study found that the prediction result of the interpolation method is consistent with the data set, that is, the data set is reliable. This map is compared with the age-based height map of Chinese children and adolescents. From the perspective of growth trends, the map is consistent with the growth and development of children and adolescents. From the perspective of the prediction results, the lifetime height predicted by the map is more accurate, so the height map based on bone age has more practical reference value. It is verified by the return visit data of the Bone Age Research Center, which is superior to traditional prediction methods. and explains the feasibility of the height growth trend map based on bone age proposed in this paper. Using this method to predict height can not only predict height based on the group law but also calculate the continuous height value before skeletal age, which has practical value in the process of medical diagnosis.

The growth trend map of children and adolescents proposed in this paper is based on the samples from the Zhejiang primary and secondary school students, so it has a high accuracy rate for children and adolescents in Zhejiang Province, but still has some errors for students from other province. In future work, we need to expand the scope of our sample collection to create a growth trend map with a larger scope of application.

## Figures and Tables

**Figure 1:** Polynomial fit map of boys based on bone age growth trend. (a) Linear function fitting; (b) quadratic function fitting; (c) cubic function fitting; (d) quartic function fitting.

**Figure 2:** Polynomial fit map of girls based on bone age growth trend. (a) Linear function fitting; (b) quadratic function fitting; (c) cubic function fitting; (d) quartic function fitting.

**Figure 3:** Height growth trend map of boys and girls based on bone age after fitting. (a) Boys' bone age height growth trend; (b) girls' bone age height growth trend.

**Figure 4:** Growth trend map based on bone age prediction. (a) Boys' predicted height growth trend; (b) girls' predicted height growth trend.

**Figure 5:** Growth trend map based on age prediction (a) Boys' predicted height growth trend (b) Girls' predicted height growth trend.

**Figure 6:** Growth trend map comparison based on age and bone age. (a) Boys' predicted height growth comparison; (b) girls' predicted height growth comparison.

**Algorithm 1:** Individual growth trend prediction algorithm.

**Table 1:** Table of height percentiles for boys in primary and secondary schools in Zhejiang based on bone age (unit: cm).

Bone age (year)	Sum of samples	3^rd^	25^th^	50^th^	75^th^	97^th^
6	254	108.2	113.3	117.1	120.3	126.6
6.5	509	109.7	115.2	118.8	122.0	129.0
7	843	113.2	118.1	121.4	124.4	130.0
7.5	1084	114.1	120.1	123.5	126.8	134.0
8	1013	116.3	122.9	126.4	130.0	135.9
8.5	1326	119.9	126.2	130.1	133.4	140.3
9	670	123.0	129.3	133.1	136.9	143.6
9.5	652	124.2	131.0	135.1	138.2	145.5
10	1119	127.9	133.7	137.4	141.1	148.0
10.5	629	130.9	136.9	141.0	144.4	152.0
11	464	132.7	139.2	142.6	146.3	153.3
11.5	735	134.9	140.1	144.1	147.6	154.2
12	855	137.3	143.6	146.9	151.2	158.2
12.5	819	139.6	146.1	150.1	154.2	162.2
13	566	144.7	150.2	155.1	159.4	167.4
13.5	407	146.6	153.3	158.2	163.1	170.1
14	448	150.4	157.3	161.7	166.5	174.1
14.5	227	156.7	163.5	166.7	170.2	178.4
15	74	159.2	165.9	168.5	172.1	181.5
15.5	46	162.3	168.4	170.2	173.9	182.8
16	53	164.9	170.1	172.1	175.2	184.4
16.5	55	165.9	171.1	173.0	176	184.4
17	53	166.3	171.6	173.6	176.6	184.7
17.5	47	166.7	171.9	173.9	176.9	185.0
18	45	166.9	172.1	174.1	177.2	185.4

**Table 2:** Table of height percentiles for girls in primary and secondary schools in Zhejiang based on bone age (unit: cm).

Bone age (year)	Sum of samples	3^rd^	25^th^	50^th^	75^th^	97^th^
5.5	123	105.5	111.4	114.3	116.8	123.9
6	375	109.6	113.2	116.5	119.3	126.6
6.5	570	110.3	115.3	118.6	121.7	127.0
7	792	112.4	118.2	121.0	124.3	129.7
7.5	804	114.6	120.5	123.7	126.9	132.9
8	775	116.7	123.0	126.2	129.6	135.8
8.5	617	118.5	124.2	128.1	131.5	138.5
9	924	121.2	127.0	130.8	134.5	141.6
9.5	1104	125.4	131.4	135.5	138.9	145.2
10	358	128.8	134.2	138.1	141.9	147.8
10.5	725	129.4	136.2	140.2	144.3	151.7
11	658	134.1	140.1	143.9	147.4	155.2
11.5	740	135.8	142.8	146.9	150.9	157.7
12	905	140.7	146.4	150.0	154.4	162.2
12.5	587	144.1	149.7	153.3	157.8	164.2
13	364	145.3	151.0	154.7	158.5	167.1
13.5	363	147.1	152.2	156.1	160.6	168.7
14	231	148.0	153.1	156.8	161.3	170.2
14.5	126	150.5	155.2	158.6	162.4	171.4
15	115	151.2	156.4	159.1	163.1	172.2
15.5	171	152.1	156.7	160.7	164.6	173.1
16	92	152.2	156.8	160.8	164.8	173.2
16.5	65	152.5	157.1	161.3	165	173.5
17	70	152.7	157.3	161.5	165.4	173.8
17.5	73	152.9	157.5	161.7	165.6	174

**Table 3:** Basic growth and development of boys.

	2011/10/23	2012/11/7	2019/4/2
Bone age/year	12.3	13.6	—
Age/year	11.5	12.5	—
Height/cm	145	154	173

**Table 4:** Basic growth and development of girls.

	2013/7/15	2014/10/18	2019/4/11
Bone age/year	12	13.4	—
Age/year	13.5	14.7	—
Height/cm	155.8	164	166

## Data Availability

The data set used to support the findings of this study was supplied by the Zhejiang Provincial Bone Age Research Center in China, under license, and the data set involving privacy cannot be shared.
